The article "Aerobics Image Classification Algorithm Based on Modal Symmetry Algorithm" was published in 2021. Journal: Comput Intell Neurosci.

# Aerobics Image Classification Algorithm Based on Modal Symmetry Algorithm

**DOI:** 10.1155/2021/5970957

**Published:** 2021-09-03

**Authors:** Xiaohua Chen, Qiang Sheng, Bhupesh Kumar Singh

**Affiliations:** ^1^Sports Department, Henan Medical College, Zhengzhou 451191, China; ^2^Arba Minch Institute of Technology, Arba Minch University, Arba Minch, Ethiopia

## Abstract

There exist large numbers of methods/algorithms which can be used for the classification of aerobic images. While the current method is used to classify the aerobics image, it cannot effectively remove the noise in the aerobics image. The classification time is long, and there are problems of poor denoising effect and low classification efficiency. Therefore, the aerobics image classification algorithm based on the modal symmetry algorithm is proposed. The method of nonlocal mean filtering based on structural features is used to denoise the aerobics image, and the pyramid structure of the image is introduced to decompose the aerobics image. According to the denoising and decomposition results, the enhancement of aerobics image is realized by the logarithmic image processing (LIP) model and gradient sharpening method. Finally, the aerobics image after the enhancement is classified by a modal symmetry algorithm. Experimental results show that the proposed method has a good denoising effect and high classification efficiency, which shows that the algorithm has significant effectiveness and high application performance.

## 1. Introduction

Classification of the image is one of the main aspects of digital image processing. It starts in the late 1950s and has been extensively used in various fields like human-car tracking, geology, climate detection, monitoring of natural calamities, medical, communications, military, and other fields of engineering [1–4]. Digital image processing is an important branch of information technology, including image denoising, enhancement, restoration, segmentation, and feature extraction [5, 6]. With the development and popularization of computer technology, the demand for digital images in agriculture, animal husbandry, forestry, environment, military, industry, and medicine is also growing. It can be said that image processing technology has penetrated into all aspects of our lives [7–9]. At present, some people are in subhealth state, and more and more people pay attention to physical exercise. Aerobics is a relatively simple and popular sport, which is widely concerned. In the process of aerobics teaching, decomposition teaching is essential, and the performance of decomposition action image recognition has a direct impact on the effect of aerobics teaching. Therefore, the aerobics image classification method has become the focus of current research. At present, there are some problems in aerobics image classification, such as poor denoising effect and low classification efficiency, so it is necessary to study the aerobics image classification method [10, 11].

Zhao and Feng put forward the aerobics image classification algorithm based on sparse coding and spatial pyramid matching. This algorithm sparse encodes the SIFT features of aerobics image, instead of the traditional vector quantization method, which can effectively reduce the quantization error and build a more accurate image representation. Then, combined with the spatial pyramid matching algorithm, the linear classifier is used for aerobics image classification and recognition. The algorithm takes a long time to sparse code SIFT features, resulting in a long time to classify, so there is a problem of low classification efficiency [12]. Shen et al. [13] put forward the aerobics image classification algorithm based on edge detection. This algorithm preprocesses the aerobics image, including image denoising and image enhancement. The region of interest in the aerobics image is obtained by the edge detection method, and the features of the detected region of interest are extracted by a gray level cooccurrence matrix. For the extracted features, a support vector machine is used for classification. After denoising, the image signal frequency fluctuates greatly, which indicates that the denoising effect of the algorithm is poor. Lu et al. [14] have proposed the aerobics image classification algorithm based on feature optimization. This algorithm carries on the threshold segmentation, the morphological filtering, and the edge tracking to the collected aerobics image to obtain the complete color back image. At the same time, based on the image set to extract the texture features, combined with the F-score feature evaluation method, the feature parameters are selected as the optimal feature subset, which is used as the input feature value of the BP neural network to realize the classification of aerobics image. This algorithm takes a long time to screen the feature parameters and has the problem of low classification efficiency. Zhao et al. [15] put forward the aerobics image classification algorithm based on the adaptive soft distribution of synonyms and chi-square model. The algorithm uses the probability latent semantic analysis model to analyze the semantic symbiosis probability of visual words in the image, excavates the hidden semantic subject of the image, and then obtains the probability distribution of the semantic subject on a visual word. The K-L divergence is introduced to measure the semantic correlation between visual words and acquire semantic related synonyms. The soft mapping between SIFT feature points and some semantic related synonyms is realized by combining the adaptive soft allocation strategy. The chi-square model is used to filter out “visual stop words” and reconstruct the histogram of visual word distribution and an SVM classifier is used to complete the target classification. This algorithm cannot effectively remove the noise in the aerobics image, and there is a problem of poor denoising effect. So based on the literature, it is found that most of the available methods cannot effectively remove the noise in the aerobics image. The classification time is long, and there are problems of poor denoising effect and low classification efficiency. Therefore, the aerobics image classification algorithm based on the modal symmetry algorithm is proposed. The results of the proposed model are better than the other currently available methods.

To sum up, this paper puts forward the aerobics image classification algorithm based on the modal symmetry algorithm. The specific process is as follows:

1. The aerobics image is denoised
2. The aerobics image then undergoes enhancement processing
3. The classification of aerobics sports image is realized by modal symmetry algorithm
4. Experiments and discussion: the overall effectiveness of the aerobics image classification algorithm based on modal symmetry algorithm is verified in two aspects of denoising effect and classification efficiency
5. Conclusions

## 2. Preprocessing of Aerobics Images

### 2.1. Nonlocal Mean Filtering Based on Structural Features

The basic features of gray image mainly include gray value, edge, texture, geometry, and spatial relationship of image. The target features extracted by the aerobics image classification algorithm based on the modal symmetry algorithm include the local edge, shape, special point, and special line of the pixel which represent the local structure of the image. To some extent, these local features can reflect the most important and essential feature information in the image [16, 17].

The denoising process of aerobics image classification algorithm based on modal symmetry algorithm is as follows:

(1) Input noise image and reduce its sensitivity to noise with Gaussian filter.
(2) Each pixel block is represented by a binary descriptor.
In order to facilitate the calculation, a set of specific neighborhood pixels is selected to represent the feature information of the central block, measure the similarity, and screen the feature similar blocks. Local block matching can also be measured by the distance between the central block and the selected reference block in its neighborhood by using the following equation:
  (1) $$\begin{array}{c} {\text{d}}_{p,q\left(m\right)}^{2}\left(B\left(p,f\right),B\left(q\left(m\right),f\right)\right)=\frac{1}{{\left(2f+1\right)}^{2}}\sum_{j\in B\left(0,f\right)}{\left(s_{p+j}-s_{q\left(m\right)+j}\right)}^{2}. \end{array}$$
Before the start, the image is smoothed by the Gaussian filter to reduce its sensitivity to noise. *s*_*p*+*j*_ and *s*_*q*(*m*)+*j*_ represent the pixel values corresponding to the center block and the neighborhood block in the smoothed image. The neighborhood block used to represent the feature information is preselected according to the experimental data, and *q*(*m*) is the *m*-the preselected neighborhood block.
 To facilitate calculation, if the local distance is less than a certain threshold *T*_1_, it means that the central pixel block is relatively flat and has no obvious structural features, and then, its binary string is directly set to 0 as given in
  (2) $$\begin{array}{c} \tau_{p}≔0,\text{if }\max\left({\text{d}}_{p,q\left(m\right)}^{2}\right)<T_{1}, \end{array}$$
where max(d_*p*,*q*(*m*)_^2^) represents the maximum value in d_*p*,*q*(*m*)_^2^.
 If max(d_*p*,*q*(*m*)_^2^) is greater than *T*_1_, it means that the central pixel block contains local image feature information; then its binary string is defined as given in
  (3) $$\begin{array}{c} \tau_{p}\left(m\right)≔\left\{\begin{array}{cc} 1, & \text{if }{\text{d}}_{p,q\left(m\right)}^{2}<{\text{d}}_{p,q\left(m-1\right)}^{2}\text{ and }{\text{d}}_{p,q\left(m\right)}^{2}\leq {\text{d}}_{p,q\left(m-1\right),}^{2}\\ 0, & \text{otherwise,} \end{array}\right. \end{array}$$
where *τ*_*p*_(*m*) represents the *m*-th bit in the string. The local distance is less than the local distance of the adjacent two pixel blocks; that is, the center point of the block that is more like the center block than the adjacent two pixel blocks is recorded as 1; the rest is 0, where d_*p*,*q*(0)_ to d_*p*,*q*(15)_ are considered as an annular. From the above definition, it can be concluded that the local binary descriptor is a 16-bit binary code and can better describe the local characteristics of pixels [18]. The binary descriptors of local similar blocks can be distinguished from other nonsimilar blocks quickly.
(3) Generate corresponding binary descriptor template for each binary descriptor to match.
 Binary descriptors can effectively improve the matching efficiency of similar blocks by comparing the binary codes (*τ*_*p*_ and *τ*_*q*_) of central pixel block and neighboring pixel block. However, in order to improve the denoising effect, more similar blocks should be selected to avoid information loss. The aerobics image classification algorithm based on the modal symmetry algorithm adopts a new local binary feature descriptor template to select more similar blocks through logical operation [19].
 Let the coding of the central pixel block be $\tau_{p}=\left[\begin{array}{cccc} 0000 & 1000 & 0000 & 0100 \end{array}\right]$, and let the coding of the two preselected similar blocks located in *q*_1_ and *q*_2_ be $\tau_{q_{1}}=\left[\begin{array}{cccc} 0000 & 1000 & 0000 & 1000 \end{array}\right]$ and $\tau_{q_{2}}=\left[\begin{array}{cccc} 0000 & 0010 & 0000 & 0001 \end{array}\right]$, respectively. In order to retain more feature information, the coding *τ*_*p*_ of the original central pixel block *p* is extended so that the left and right binary numbers with the coding median value of 1 are also 1, and the descriptor *τ*_*p*_′ is obtained by using
  (4) $$\begin{array}{c} \tau_{p}^{\prime }\left(m\right)≔1,\;\text{if }\tau_{p}\left(m-1\right)=0,\text{or }\tau_{p}\left(m+1\right)=1,\text{ or }\tau_{p}\left(m\right)=1. \end{array}$$
 After that, the descriptor template and its coding of neighborhood pixel block are made bit operation. If the result is equal to the neighborhood coding, it is regarded as similar to the central pixel block; otherwise, it is not similar and can be represented as follows [20]:
  (5) $$\begin{array}{c} \left\{\begin{array}{cc} \left(\tau_{p}^{\prime }\&\tau_{q}\right)=\tau_{q}, & \text{similar,}\\ \left(\tau_{p}^{\prime }\&\tau_{q}\right)\neq \tau_{q}, & \text{not similar.} \end{array}\right. \end{array}$$
(4) For a pixel block whose binary descriptor is greater than 0, it means that the region contains characteristic information. Then,
  (1) Features and gray similar blocks are selected by the following prescreening equation:
    (6) $$\begin{array}{c} B_{p}-B_{q}|<k\times \sigma_{n}. \end{array}$$
  (2) The corresponding weights of similar blocks can be calculated by the following equation:

(7) $$\begin{array}{c} \left\{\begin{array}{cc} w_{k,l}=1, & {\text{d}}_{k,l}^{2}\leq T_{1},\\ w_{k,l}=\frac{\left(T_{2}-{\text{d}}_{k,l}^{2}\right)}{\left(T_{2}-T_{1}\right)}, & T_{1}<{\text{d}}_{k,l}^{2}\leq T_{2},\\ w_{k,l}=0, & {\text{d}}_{k,l}^{2}>T_{2}, \end{array}\right. \end{array}$$

where d_*k*,*l*_^2^ is the Euclidean distance between the center pixel block *u*_*i*,*j*_^*N*_*p*_^ and the preselected similar block *u*_*k*.*l*_^*N*_*p*_^. It can be calculated using

(8) $$\begin{array}{c} {\text{d}}_{k,l}^{2}=\frac{{\left\|u_{k.l}^{N_{p}}-u_{i,j}^{N_{p}}\right\|}_{2}^{2}}{{\left(2N_{p}+1\right)}^{2}},\;\forall k,l\in \Omega_{i,j}^{N_{s}}, \end{array}$$

where *N*_*p*_ represents the size of the pixel block, and the thresholds *T*_1_ and *T*_2_ are defined by the following equation:

(9) $$\begin{array}{c} \left\{\begin{array}{c} T_{1}=\lambda \sigma_{n}^{2},\\ T_{2}=2T_{1}. \end{array}\right. \end{array}$$

### 2.2. Image Enhancement

#### 2.2.1. Image Pyramid

For an image *M* with *N* × *N*(*N*=2^*n*^), 1/2 subsampling in two directions can obtain a 1/4 thumbnail of the original image. Through continuous subsampling, we can get a series of pyramid structures composed of subimages of different sizes, and each layer of which has different sizes and resolutions. The size of layer 0 is the largest and the resolution is the highest. With the movement to the upper layer of the pyramid, the size and resolution of the image decrease until layer *n* [21].

In the process of building the pyramid, from the later level to the former level, the resolution of the row and column is reduced by factor 2, and the size of the image is reduced accordingly. For a complete two-dimensional image pyramid with *n*+1 layers in total, the total number of elements is given by

(10) $$\begin{array}{c} N^{2}\left(1+\frac{1}{4}+\frac{1}{4^{2}}+\cdots \right)\leq \frac{4}{3}N^{2}. \end{array}$$

The low-scale level mainly shows the contour information of the image, while the high-scale level reflects the detail characteristics of the image [22].

Only depending on subsampling to reduce the size of the image, we often lose a lot of information. According to the sampling theorem, it is necessary to make all the images obtained by sampling at the shortest wavelength less than 1/4 pass the smoothing filter to eliminate the distortion. From the perspective of scale space, reducing image size needs to be synchronized with appropriate image smoothing filtering. If smoothing and subsampling are repeated, subimages with different resolutions can be obtained [23, 24]. The image pyramid can be formed by sorting the obtained subimages.

Taking the Gaussian pyramid as an example, the Gaussian low-pass smoothing filtering process can be expressed as *R*(*x*, *y*, *σ*) and can be found by

(11) $$\begin{array}{c} R\left(x,y,\sigma \right)=G\left(x,y,\sigma \right)\times I\left(x,y\right). \end{array}$$

That is to say, the two-dimensional image *I*(*x*, *y*) is convoluted with the Gaussian filter *G*(*x*, *y*, *σ*) to obtain the smoothed image *R*(*x*, *y*, *σ*), where the expression of the Gaussian filter *G*(*x*, *y*, *σ*) is as follows:

(12) $$\begin{array}{c} G\left(x,y,\sigma \right)=\frac{1}{2\pi \sigma^{2}}e^{-x^{2}+y^{2}/2\sigma^{2}}. \end{array}$$

The scale parameter is the bandwidth *σ* of the Gaussian filter. Using Gaussian smoothing filter, the single operation *G*^(*k*+1)^ of generating Gaussian pyramid subimage can be expressed as follows:

(13) $$\begin{array}{c} G^{\left(k+1\right)}=S_{\left(↓2\right)}G^{\left(k\right)}. \end{array}$$

That is to say, the *k*-th layer Gaussian image *G*^(*k*)^ is used to calculate the *k*+1-th layer Gaussian image *G*^(*k*+1)^, where *S* represents the Gaussian smoothing operator and its subscript (↓2) represents subsampling with a sampling rate of 2. The bottom layer of the pyramid is the original image, and the highest layer corresponds to the thickest size.

#### 2.2.2. Enhancement Algorithm of the LIP Model

The enhancement algorithm based on the LIP model simplifies the gray-scale image by using the unified complement transformation. The simplified processing algorithm of gray-scale function is expressed in the form of

(14) $$\begin{array}{c} f{}^{\prime }=1-\frac{f}{m}, \end{array}$$

where *f*′ represents the output image after the normalization and complement transformation, and the value range of the gray function *f* is defined in interval [0, *m*] for nonlinear transformation as expressed in

(15) $$\begin{array}{c} \ln\left[f^{1}\left(i,j\right)\right]=\alpha \;\ln\left[f{}^{\prime }\left(i,j\right)\right]+\beta \;\ln\left\{f{}^{\prime }\left(i,j\right)-\ln\left[a{}^{\prime }\left(i,j\right)\right]\right\}, \end{array}$$

where *f*′(*i*, *j*) and *f*^1^(*i*, *j*) are input and output pixel gray values, *α* and *β* are real numbers respectively, and the expression of ln[*a*′(*i*, *j*)] is as follows:

(16) $$\begin{array}{c} \ln\left[a{}^{\prime }\left(i,j\right)\right]=\frac{1}{{\left(n+1\right)}^{2}}\sum_{k=i-n/2}^{i+n/2n/2}\sum_{l=j-n/2}^{j+n/2}\ln\left[f{}^{\prime }\left(k,l\right)\right]. \end{array}$$

When 0 < *α* < 1, the nonlinear transformation process can expand the dynamic range of the dark area of the image. When *α* > 1, the process can expand the dynamic range of the bright area of the image. When *β* > 1, the difference between the mean value of the central pixel and the surrounding pixel is magnified nonlinearly. The larger the *β* value is, the greater the edge enhancement of the image is.

#### 2.2.3. Gradient Sharpening

Gradient algorithm is used to sharpen image edge information. The gradient of the function *f*(*x*, *y*) at a point (*x*, *y*) is defined as a vector as

(17) $$\begin{array}{c} G\left[f\left(x,y\right)\right]=\left(\frac{\partial f}{\partial x},\frac{\partial f}{\partial y}\right). \end{array}$$

That is, the direction of the gradient is in the direction of the maximum change rate of function *f*(*x*, *y*), and the magnitude of the gradient is defined as given by

(18) $$\begin{array}{c} G{}^{\prime }\left[f\left(x,y\right)\right]=\sqrt{{\left(\frac{\partial f}{\partial x}\right)}^{2}+{\left(\frac{\partial f}{\partial y}\right)}^{2}}. \end{array}$$

A threshold *T* is introduced to determine whether to process the gray value of a pixel, which is given by

(19) $$\begin{array}{c} G\left(i,j\right)=\left\{\begin{array}{cc} A, & G\left[f\left(i,j\right)\right]>T,\\ 0, & G\left[f\left(i,j\right)\right]\leq T. \end{array}\right. \end{array}$$

The gradient value between the background and the object does not change much. The obvious change of gray level is mainly reflected in the junction of the object and the background, that is, the edge of the image. By setting the threshold value, *G*[*f*(*i*, *j*)] of the image edge's gray value is greater than the threshold value, which makes the pixel point bright and highlights the edge; for the same pixel gray value *G*[*f*(*i*, *j*)] is not greater than the threshold value, it is smoothed [25, 26].

## 3. Aerobics Image Classification Algorithm Based on Modal Symmetry Algorithm

The aerobics image classification algorithm based on the modal symmetry algorithm realizes the aerobics image classification through the modal symmetry algorithm. The specific steps are as follows.

### 3.1. Establishing “Visual Vocabulary”

Supposing that we train a MIL classifier for a scene *C*, let *L*={(*B*_1_, *y*_1_), (*B*_2_, *y*_2_),…, (*B*_*N*_, *y*_*N*_)} denote the labeled image set, where *y*_*i*_ ∈ {−1, +1}, *i*=1,2,…, *N*+1 denotes the image belonging to scene *C*, −1 denotes the image not belonging to scene *C*, and *Q*={*B*_1_, *B*_2_,…, *B*_*M*_} denotes the unlabeled image set. If any image *B* is divided into *n*_*i*_ regions, the corresponding visual feature vector of each region is recorded as *X*_*ij*_ ∈ *R*^*d*^, *j*=1,2,…, *n*_*i*_, and *d* represents the dimension of the visual feature vector, then *B*_*i*_={*X*_*ij*_*|j*=1,…, *n*_*i*_} is the MIL training package, and *X*_*ij*_ is the example in the package. All the examples of all the images in *L* are put together, called the example set, and record it as IntSet and given by

(20) $$\begin{array}{c} \text{IntSet}=\left\{X_{t}|t=1,2,\ldots ,P\right\}, \end{array}$$

where *P* is the total number of examples, and its calculation formula is as follows:

(21) $$\begin{array}{c} P=\sum_{i=1}^{N}n_{i}. \end{array}$$

The aerobics image classification algorithm based on modal symmetry algorithm uses *K*-Means method to gather the elements in IntSet into *K* class. Because each clustering center usually represents a group of image areas with the same visual characteristics, it is called a “visual word” [27], and it is recorded as *v*_*i*_, and these *K* “visual words” are called “visual vocabulary” and recorded as Ω={*v*_1_, *v*_2_,…, *v*_*k*_}.

### 3.2. Constructing Fuzzy “Word-Document” Matrix

In order to obtain the latent semantic model of the image by LSA method, according to the principle of minimum Euclidean distance, the number of different “visual words” appearing in the multiple sample packets is counted; that is, the multiple sample packets are represented by word frequency vector [28]. Let the word frequency vector of the multiple example package *B*_*j*_ be *F*_*r*_*j*__ as given in

(22) $$\begin{array}{c} F_{r_{j}}=\left[n_{1,l},n_{2,l},\ldots ,n_{K,l}\right], \end{array}$$

where *n*_*i*,*l*_ represents the number of occurrences of the *i*-th “visual word” *v*_*i*_ in *B*_*j*_. In terms of word frequency statistics, the traditional method is as follows: if the example *X* is closest to the Euclidean distance of “visual word” *v*_*i*_, then add 1 to the *i*-th component value of word frequency vector, i.e., *n*_*i*,*l*_=*n*_*i*,*l*_+1, and there is irrationality in the way of word frequency statistics. Let *v*_1_ and *v*_2_ represent two different “visual words” and *E*, *F*, *G*, and *H* represent four different examples. From Figure 1, it can be seen intuitively that the confidence of *E* is higher than that of *F* belonging to *v*_1_, while the distance between *G* and *v*_1_ and *v*_2_ is the same, and there is ambiguity in whether *G* belongs to *v*_1_ or *v*_2_. Traditional word frequency statistical methods do not consider these differences and ambiguity [29].

To solve this problem, the fuzzy membership function *f*=*f*(*X*, *v*)=exp(−‖*X* − *v*‖^2^) is defined according to the Euclidean distance between example *X* and “visual word” *v*. It can be said that each example in the multiexample package belongs to all the “visual words” at the same time; only according to the distance, the degree of membership is different. Through the above analysis, the fuzzy word frequency vector defined by the aerobics image classification algorithm based on the modal symmetry algorithm can be represented by

(23) $$\begin{array}{c} \left\{\begin{array}{c} S_{j}=\left[s_{1,j},s_{2,j},\ldots ,s_{K,j}\right],\\ s_{i,j}=\sum_{t=1}^{n_{j}}f\left(X_{jt},v_{i}\right)=\sum_{t=1}^{n_{j}}\exp\left(-{\left\|X_{jt}-v_{i}\right\|}^{2}\right), \end{array}\right. \end{array}$$

where *X*_*jt*_ represents the *t*-th example in the multisample package *B*_*j*_ and *n*_*j*_ represents the number of examples in *B*_*j*_. It can be seen from the above formula that the value *s*_*i*,*j*_ of the *i*-th component of the fuzzy word frequency vector is determined by the sum of the fuzzy membership degrees between all the examples in *B*_*j*_ and *v*_*i*_ [30].

In order to highlight the importance of different “visual words” in image classification, the fuzzy word frequency vector is weighted by word frequency-anti-document frequency, namely,

(24) $$\begin{array}{c} w_{i,j}=s_{i,j}\times 1b\left(1+\frac{N}{\text{d}f_{i}}\right), \end{array}$$

where *s*_*i*,*j*_ represents the fuzzy frequency of *B*_*j*_ containing “visual word” *v*_*i*_; d*f*_*i*_ represents the number of multiple sample packets containing “visual word” *v*_*i*_ in the training set; *N* represents the total number of all multiple sample packets in the training set.

In order to control the change range of *w*_*i*,*j*_ within the same range, normalization is carried out, as given by

(25) $$\begin{array}{c} {\bar{w}}_{i,j}=\frac{w_{i,j}}{\sum_{i=1}^{K}w_{i,j}}. \end{array}$$

The weighted and normalized word frequency vector is recorded as $W_{j}=\left[{\bar{w}}_{1,j},{\bar{w}}_{2,j},\ldots ,{\bar{w}}_{K,j}\right]$. By arranging the fuzzy word frequency vectors corresponding to all multiple example packages in the training set, we can get the fuzzy “word-file” knowledge matrix, which is recorded as given by

(26) $$\begin{array}{c} A_{K\times N}=\left[W_{1},W_{2},\ldots ,W_{N}\right]=\left[\begin{array}{cccc} {\bar{w}}_{1,1} & {\bar{w}}_{1,2} & \ldots & {\bar{w}}_{1,N}\\ {\bar{w}}_{2,1} & {\bar{w}}_{2,2} & \ldots & {\bar{w}}_{2,N}\\ \ldots & \ldots & \ldots & \ldots \\ {\bar{w}}_{K,1} & {\bar{w}}_{K,2} & \ldots & {\bar{w}}_{K,N} \end{array}\right], \end{array}$$

where each row of *A*_*K*×*N*_ corresponds to a “visual word” and each column corresponds to a multiple sample package.

### 3.3. Fuzzy Latent Semantic Features

As a natural language processing method, LSA's core idea is to build a potential semantic space through truncated singular value decomposition and project words and documents to various dimensions representing potential semantics, so that the potential semantic relationship between words can be obtained, and the related documents can obtain the same vector representation even if they do not use the same words [31, 32]. According to the singular value decomposition theorem, the matrix *A*_*K*×*N*_ of “word-file” can be decomposed into three matrix products, as given by

(27) $$\begin{array}{c} A_{K\times N}=U_{K\times n}D_{n\times n}\left(V_{N\times n}\right), \end{array}$$

where *K* is the dimension of the original feature space, *n*=min(*K*, *N*), *U* and *V* are left and right singular vector matrices corresponding to the singular value of matrix *A*, respectively, and *U*′*U*=*V*′*V*=*I* and *D* are diagonal matrices which arrange the singular value of matrix *A* in descending order. If only the first *T* singular values in *D*_*n*×*n*_ and the first *T* columns of *U*_*K*×*n*_ and *D*_*n*×*n*_ are taken, that is, *U*_*K*×*T*_, *D*_*T*×*T*_, and *V*_*N*×*T*_, then the best approximation of matrix *A*_*K*×*N*_ in the sense of *T*-order least squares can be obtained, as given by

(28) $$\begin{array}{c} A_{K\times N}^{\prime }=U_{K\times T}D_{T\times T}V_{N\times T}. \end{array}$$

In general, the above formula is called truncated singular value decomposition. In this way, the matrix after dimension reduction of *A*_*K*×*N*_ can be obtained; that is, ${\bar{A}}_{T\times N}=D_{T\times T}V_{N\times T}$. Here, each column in ${\bar{A}}_{T\times N}$ is the fuzzy latent semantic feature of the corresponding package in the training set, which is reduced from the original *K* dimension to the *T* dimension. Let $W=\left[{\bar{w}}_{1},{\bar{w}}_{2},\ldots ,{\bar{w}}_{K}\right]$ be the normalized fuzzy word frequency vector of any new multiexample package *B*, and its fuzzy latent semantic features are as given by

(29) $$\begin{array}{c} \phi \left(B\right)=\left(U_{K\times T}\right){}^{\prime }W. \end{array}$$

This is derived from *A*=*UDV*′⇒*U*′*A*=*U*′*UDV*′⇒*U*′*A*⇒*DV*′, where the space formed by *T* column vectors in *U*_*K*×*T*_ is called fuzzy latent semantic space, which can be regarded as the compression of the original vector space. *T* column vectors in *U*_*K*×*T*_ are the basis of fuzzy latent semantic space.

### 3.4. Training TSVM Classifier (*w*^*∗*^)

*TS* ≠ ∅ is initialized, ∀*B*_*j*_ ∈ *L* is as labeled package, and its fuzzy latent semantic feature *ϕ*(*B*_*i*_) is calculated; then (*ϕ*(*B*_*i*_), *y*_*i*_) is added to TS, where *y*_*i*_ is the label of package *B*_*i*_. If ∀*B*_*j*_ ∈ *Q* is an unmarked package, its fuzzy latent semantic feature ∀*B*_*j*_ ∈ *Q* is calculated. (*ϕ*(*B*_*j*_^*∗*^), *y*_*i*_) is added to TS, where the label of the unmarked package is 0.

The TS is used to solve the following optimization problem, and the class label {*y*_*j*_^*∗*^}_*j*=1_^*M*^ ∈ {−1, +1} and the TSVM classifier (*w*^*∗*^) of the unlabeled image set *Q* are obtained as given by

(30) $$\begin{array}{c} \left\{\begin{array}{cc} \min\left(w,y_{1}^{*},\ldots ,y_{M}^{*}\right): & \frac{\lambda }{2}{\left\|w\right\|}^{2}+\frac{1}{2N}\sum_{i=1}^{N}\text{los}\left[y_{i}w^{T}\phi \left(B_{i}\right)\right]+\frac{\lambda^{*}}{2M}\sum_{j=1}^{M}\text{loss}\left(y_{j}^{*}w^{T}\right)\phi \left(B_{j}^{*}\right),\\ \text{subject to}: & \frac{1}{M}\sum_{j=1}^{M}\max\left[0,\text{sign}\left(w^{T}\phi \left(B_{j}^{*}\right)\right)\right]=r, \end{array}\right. \end{array}$$

where *M* is the total number of unlabeled samples; loss(*z*) is the loss function, usually loss(*z*)=max(0,1 − *z*); *y*_*j*_^*∗*^ ∈ {−1,1}; *M* is the label assigned to unlabeled samples in the optimization process; *r* is the proportion of the number of samples to be marked as positive in the total number of unlabeled samples; and the control parameter *λ* is used to adjust the balance between algorithm complexity and loss function.

Through the above process, the classification of aerobics sports image is achieved.

## 4. Experiment and Discussion

In order to verify the overall effectiveness of the aerobics image classification algorithm based on the modal symmetry algorithm, it is necessary to test the aerobics image classification algorithm based on the modal symmetry algorithm. This test is completed in the MATLAB platform. The aerobics image classification algorithm based on the modal symmetry algorithm (algorithm 1), the aerobics image classification algorithm based on the sparse coding space pyramid matching (algorithm 2), the aerobics image classification algorithm based on edge detection (algorithm 3), and the aerobics image classification algorithm based on feature optimization (algorithm 4) are used to test. The above algorithms are used to denoise the aerobics image, and the signal frequency of the image before and after denoising is compared with four different methods. The test results are as represented in Figure 2.

Figure 2 represents the comparison of the image signal frequency before and after denoising by four different algorithms. It can be seen that the signal frequency after denoising of aerobics image classification algorithm based on modal symmetry algorithm is smaller than that before denoising for all the iterations. The more the denoising effect is, the more suitable the algorithm is to achieve a stable frequency. The signal frequency tends to be stable, indicating that the aerobics image classification algorithm based on modal symmetry algorithm has a good denoising effect because the algorithm uses a new local binary feature descriptor template to filter out more similar blocks through logical operation to avoid information loss and improve the denoising effect.

The aerobics image classification algorithm based on modal symmetry algorithm (algorithm 1), the aerobics image classification algorithm based on sparse coding space pyramid matching (algorithm 2), the aerobics image classification algorithm based on edge detection (algorithm 3), and the aerobics image classification algorithm based on feature optimization (algorithm 4) are tested, respectively, the classification times of four different algorithms are compared, and the test results are as follows.

The analysis of Figure 3 shows that the classification time of aerobics image classification algorithm based on modal symmetry algorithm in multiple iterations is lower than that of aerobics image classification algorithm based on sparse coding space pyramid matching, the aerobics image classification algorithm based on edge detection, and the aerobics image classification algorithm based on feature optimization because the aerobics image classification algorithm based on the modal symmetry algorithm enhances the aerobics image between the classification, improves the significance of the image characteristics, shortens the time of classifying the aerobics image, and improves the classification efficiency of the aerobics image classification algorithm based on the modal symmetry algorithm.

## 5. Analysis

There are a number of methods and algorithms to classify the aerobic images. Most of them are slow for detection. So, it is necessary to test the aerobics image classification algorithm based on the modal symmetry algorithm. The aerobics image classification algorithm based on the modal symmetry algorithm (algorithm 1), the aerobics image classification algorithm based on the sparse coding space pyramid matching (algorithm 2), the aerobics image classification algorithm based on edge detection (algorithm 3), and the aerobics image classification algorithm based on feature optimization (algorithm 4) are used to test. The test results represented in Figure 2 indicate that the proposed method has the best denoising effect as compared to the other three methods. Also, Figure 3 shows that the proposed method has the least processing time among the four methods to denoise the aerobic images.

## 6. Conclusions

In order to classify and recognize the aerobics image, it is necessary to study the aerobics image classification algorithm. At present, the aerobics image classification algorithm has the problems of poor denoising effect and low classification efficiency. The aerobics image classification algorithm based on the modal symmetry algorithm is proposed, which can effectively remove the noise in the aerobics image in a short time, complete the classification of the aerobics image accurately, solve the problems in the current method, and provide the relevant information for the aerobics image recognition. The results presented in the results and discussion section clearly indicated that the proposed algorithm has a more denoising effect, as compared to the other methods. Also, for the proposed method, the time taken for processing data is the minimum. Hence, it is concluded that the proposed method is better than the other three methods.

## Figures and Tables

**Figure 1:** Fuzzy relationship between example and “visual word.”

**Figure 2:** Denoising results of four different algorithms. (a) Algorithm 1. (b) Algorithm 2. (c) Algorithm 3. (d) Algorithm 4.

**Figure 3:** Classification time of four different algorithms. (a) Algorithm 1 and algorithm 2. (b) Algorithm 3 and algorithm 4.

## Data Availability

Data will be made available on request to the corresponding author.
